RETRACTED

# Preparation and Sound Insulation Performance of Polystyrene Building Flame Retardant and Thermal Insulation Building Materials

**DOI:** 10.1155/2022/6444367

**Published:** 2022-06-24

**Authors:** Qiulan Guo

**Affiliations:** College of Architectural Engineering, Xinyu University, Xinyu, Jiangxi 338004, China

## Abstract

In this study, magnesium hydroxide (MH) was modified by sodium dodecylbenzene sulfonate (SDBS) to prepare modified magnesium hydroxide (MMH) flame retardant, which was mixed with polystyrene (PS) to obtain flame retardant PS composite plate. The micromorphology, mechanical properties, thermal stability, and flame retardancy of flame retardant PS composite plate were analyzed. The experimental results show that MMH is well dispersed in PS matrix, PS-MMH-3 has the best tensile strength and elongation at break, the limit oxygen index (LOI) is 44.3% higher than that of pure PS, and the combustion rate is slow, indicating that PS-MMH-3 has good flame retardant properties.

## 1. Introduction

Polystyrene foam is widely used in the fields of packaging, heat preservation, waterproof, heat insulation, shock absorption, low price because of its light weight, firmness, shock absorption, low moisture absorption, easy molding, good water resistance, heat insulation, and low price. It is one of the most widely used plastics in the world today. It can be used in the square shock packaging of electrical appliances, instruments, handicrafts, and other vulnerable valuables, as well as the packaging of fast food [1]. Waste EPS still maintains its good physical and chemical properties. It is a kind of closed hole and light thermal insulation material. Under the condition of correct construction and good waterproof, it has energy saving, good long-term R (thermal resistance), water resistance, and dimensional stability. EPS used in the field of building materials has its own advantages in the following aspects [2].

Since the 1990s, the hottest topic in the construction industry is green buildings or environment-friendly buildings. In view of the fact that many products in the market claim to be “green,” it is not easy to choose the best products for sustainable development. An important factor to consider when selecting the right insulation material is long-term performance, including thermal resistance, dimensional stability, compressive strength, insurance, and building code requirements. Some people think that traditional products have been used for decades and are definitely not green. This is not the case. EPS is a kind of green thermal insulation material before its environmental protection advantages are recognized. EPS never contains ozone depleting gases, such as CFC or HCFC. Those thermal insulation materials using CFC and HCFC are no longer in production. The original production will be reorganized to produce brand-new thermal insulation materials, and these thermal insulation materials have only short-term function tracking records [3].

RETRACTED

At present, there are three main insulation modes: internal insulation mode and external insulation mode. There are two forms of external wall insulation: insulation board and insulation mortar. At present, the insulation board is not suitable for the insulation of irregular building parts, and its application is limited due to complex construction and high comprehensive cost. However, as a new type of building material, the thermal insulation masonry mortar or block has the advantages of light weight, low thermal conductivity, low comprehensive cost, low water absorption, and convenient construction, which can overcome many shortcomings of thermal insulation board [4]. It can be seen from Figure 1 that the real significance of wall material innovation is to realize the direct self-insulation of building masonry mortar or block as soon as possible.

## 2. Literature Review

Hasheminejad used a resin as coating resin, nitrogen phosphorus chemical expansion flame retardant, and EG to make composite synergistic flame retardant, which was made into plate by molding. The effects of intercalation e.g., made of different intercalators such as perchloric acid, concentrated sulfuric acid, perchloric acid, phosphoric acid, concentrated sulfuric acid and phosphoric acid on thermal conductivity, tensile strength, oxygen index, and carbon residue rate of the composites were investigated. The EPS board is impregnated with phenolic resin and magnesite cement for flame retardant. When the concentration of magnesite cement is 15%, the oxygen index can reach 33.1% and the tensile strength is 0.189 MPa [5]. Zhang used melamine formaldehyde resin prepolymer (MF) as coating solution, ammonium polyphosphate and zinc borate as flame retardant, and EPS prefoamed particles are coated with coating solution. The experiment explored the test method and optimum process conditions for the preparation of EPS under laboratory conditions. It is found that the oxygen index of the material increases with the increase of the amount of flame retardant. When the mass ratio of EPS/MF/APP/ZB is 100/120/15/2, the LOI reaches 22.6% and the amount of carbon residue is 14.8% [6]. The method of flame retardant coating can improve the thermal shrinkage of EPS foam board, obviously slow down the combustion rate, and reduce the smoke density. Under the condition of EPS/thermosetting phenolic resin/ammonium polyphosphate in the ratio of 100/100/10 (mass ratio), He prepared polystyrene foam insulation board by the coating method. The effects of foaming temperature and foaming time on the density, compressive strength, linear expansion coefficient, and thermal conductivity of EPS beads after foaming were mainly studied. The process conditions were determined by comparison. The foaming temperature was 120°C, and the foaming time was 8 min. It is found that the oxygen index of the material increases first and then decreases with the increase of ammonium polyphosphate content. When the content of ammonium polyphosphate is 20 PHR, the horizontal combustion rate can reach FH.1 level. The study also found that the higher the content of ammonium polyphosphate, the lower the compressive strength, the higher the thermal conductivity, and the higher the linear expansion coefficient of EPS material [7]. Lu used thermosetting phenolic resin and aluminum hydroxide mixed flame retardant liquid to flame retardant cover polystyrene particles to change the combustion essence of combustion droplets and shrinkage of polystyrene insulation board. Experiments show that aluminum hydroxide (ATH) can only improve the flame retardant performance of the material in a certain range. When the ATH content exceeds a certain value, the oxygen index of the material does not increase, but decreases sharply. The experimental results show that the insulation coefficient of polystyrene insulation board prepared by flame retardant coating method is less than 0.036 w/(m K), the flame retardant performance is BL grade, and the calorific value is 20.3 MJ/kg [8]. Tian developed a flame retardant process of coating EPS with silicate, that is, EPS beads are prefoamed and cured, and then, silicate is used as inorganic flame retardant to form suspension with water, suspension (stabilizer), catalyst, expander, plasticizer, phenols, and aldehydes. The prepared suspension and EPS beads after prefoaming treatment are poured into the mold and heated for foaming [9]. Qiu mixed foaming agent powder, hardener powder, and phenolic resin powder, and then, gel treatment was carried out on the mixture of the three. Then, the mixed expandable resin powder is coated on the surface of EPS beads by spray with a nozzle. The coated EPS beads are dried with hot air; then, talc powder is added and then foamed in the mold [10]. Ovsyannikov used Freon as flame retardant, added Freon into thermosetting phenolic resin and stirred evenly to make flame retardant coating solution. The solution prepared by mixing two resins (phenolic resin and melamine resin), foaming agent, catalyst, and surfactant was mixed and stirred with EPS particles after prefoaming treatment and then put it into the mold for foaming [11]. Wang coated EPS beads with a flame retardant coating system prepared from phenolic resin, curing agent (phosphorescent agent), and phosphate ester condensed from EG and carbon forming polyol as flame retardant. Among them, dimethyl methyl phosphate, ethylene propyl 1,3-diphosphate, triethyl phosphate, diethyl ethyl phosphate, and other low viscosity aliphatic phosphoric acids or phosphate esters can be selected as flame retardants. The coating and foaming process is as follows: phosphate ester and phenolic resin are mixed into coating solution, which is mixed with EPS beads evenly and then directly heated and foamed in the mold to obtain flame retardant polystyrene foam material [12]. Tilkin coated EPS, mixed phosphate ester and carbonaceous polyol into solution, mixed with EPS beads in the mold, and then heated and foamed for integrated molding [13]. Moharana developed the coating process with triazine derivatives as flame retardants. The company adopts various alkyl substituted derivatives of 2,4 diamino 1,3,5 triazine, various alkyl substituted derivatives of 2,4,6 triamino l,3,5 triazine on nitrogen atoms, and melamine polycondensates, the most important of which is melamine. The company's invention is to conduct two coating processes on the surface of EPS beads. The outermost coating solution is a common coating solution, such as a mixture of triglyceride, glyceryl monostearate, and zinc stearate. The coating liquid of the inner layer is the coating of flame retardant [14].

RETRACTED

## 3. Experimental Part

### 3.1. Main Raw Materials

Magnesium hydroxide (MH), sodium dodecylbenzene sulfonate (SDBS), and absolute ethanol, analytical purity, were obtained from Tianjin Damao Chemical Reagent Factory. General polystyrene (PS), GP5250, was obtained from Dongguan plastic Co., Ltd. Liquid paraffin, analytical purity, was obtained from Sinopharm Chemical Reagent Co., Ltd.

### 3.2. Instruments and Equipment

Injection machine, MH-150T; contact angle tester, ZT-705SB; specific surface area tester (BET), V-Sorb 2800TP; thermogravimetric analyzer, ZRT-B; universal testing machine, WE-300B; scanning electron microscope (SEM), JSM 5900lv; oxygen index meter, YN-HC2; thermal conductivity tester, 2500-OT; UL94 vertical and horizontal combustion tester, PX-03-001; cone calorimeter, FT-5; and rotary viscometer, NDJ-79 were used [15].

### 3.3. Sample Preparation

Preparation of modified magnesium hydroxide (MMH): dry magnesium hydroxide (MH) at 100°C for 12 hours and pass through a 80-mesh sieve. Stir 1000 ml of 15% MH material in an oil bath at 90°C for 2 hours, add 15 g of SDBS, and continue stirring.

RETRACTED

Preparation of flame retardant PS composites: Table 1 provides the formula of flame retardant PS composites. Unmodified MH and MMH were mixed with PS according to the proportion in Table 1. Injection molding was carried out in the injection machine at a temperature of 195°C for 15 min. The tablet was pressed at 200°C for 20 min. After cooling, cut the sheet material into 4 cm × 3 cm×2 cm for standby [16].

### 3.4. Performance Test and Characterization

SEM Enxi: observe the surface morphology of the sample after liquid nitrogen brittle fracture and gold spraying.

TG analysis: sample 0.5 g, temperature range 25–600°C, and heating rate 10°C/min.

Contact angle test: the powder contact angle meter is used for measurement. During calculation, the contact angle without MMH is expressed as 0° as the benchmark.

Specific surface area test: the bet multipoint method is used for measurement. After vacuum degassing, the sample is placed in the cold trap and the temperature is set to 78 K.

Heat release rate test: test according to GB/T 2408–2008, heat flow 25 kW/m^2^, and sample size 20 mm × 20 mm × 20 mm.

LOI test: test according to GB/T 2408–2008, and sample size is 100 mm × 10 mm × 10 mm.

Mechanical property test: according to GB/T 14484–2008, the loading rate is 2 mm/min and the sample size is 40 mm × 30 mm × 20 mm.

Test of total heat release and smoke production: test according to GB/T 2408–2008, heat flow 20 kW/m^2^, and sample size 100 mm × 10 mm × 10 mm.

Thermal conductivity test: according to ISO 22007-2:2008, the sample size is 40 mm × 30 mm × 20 mm.

Viscosity test: prepare MH paraffin solution in different proportions and stir it fully. The test temperature is 25°C [17].

## 4. Results and Discussion

### 4.1. Property Analysis of MMH

Table 2 provides the specific surface area and water contact angle of MH before and after modification. At the same time, after MH modified grafted SDBS, due to the formation of semimicelle state, the surface transits from hydrophilicity to hydrophobicity, so the contact angle becomes larger [18].

### 4.2. Mechanical Properties of Flame Retardant PS Composite Board

Figure 2 shows the tensile strength and elongation at break of flame retardant PS composite board.

As shown in Figure 2, with the addition of MMH, the tensile strength of PS composite gradually increases, reaching the optimal value of 19.23 MPa in PS-MMH-3, and then begins to decrease. It may be because MH, as an inorganic nano particle, has high tensile strength. When blended with PS, it can improve the mechanical strength of the composite. When the content of MMH continues to increase (PS-MMH-4), inorganic nanoparticles cannot be evenly dispersed in the material, resulting in a certain agglomeration, which destroys the original structure of the polymer matrix and reduces the tensile strength to a certain extent. This is because MMH improves the compatibility in polymer matrix and can effectively improve the tensile strength of PS composite. Similar to tensile strength, the change trend of elongation at break with the increase of MH is the same as that of tensile strength, reaching the maximum value of 87% in PS-MMH-3, indicating that PS-MMH-3 has high extensibility and can be used in building materials [4, 19].

RETRACTED

### 4.3. Flame Retardant Performance of Flame Retardant PS Composite Board

The higher the LOI, the better the combustion performance of the material.  Figure 3 shows the LOI of different PS composites. As shown in Figure 4, the LOI value of pure PS is the lowest, which is 25.6%. With the addition of MMH, the LOI of the composites gradually increased and reached the peak in PS-MMH-3, and its LOI value was 44.3%. This is because MMH has high thermal stability and efficient carbon formation of substrate, which can effectively play the role of flame retardant. Grafting more organic chain hydrocarbons on MMH particles can delay the migration rate of oxygen to the interior of the material during combustion. Therefore, the LOI value is high [20].

Figure 3 shows the heat release rate (HRR) of different PS materials. It can be seen from Figure 4 that pure PS material can reach the peak heat release rate (PHRR) in a short time and terminate the heat release in a short time, indicating that its combustion process is extremely rapid. In PS-MH, due to the flame retardant effect of MH, its PHRR value is low, but it still ends the combustion process in a short time [21].  Figure 5 shows the smoke production and smoke production rate of different PS materials. As shown in Figure 5, compared with pure PS, the smoke production and smoke production rate of PS composite added with MMH are reduced. This is because the magnesium oxide layer produced by MMH during high-temperature decomposition blocks the interior of the material, thus hindering the propagation of heat. The higher the MMH content, the more heat absorption and water generated during decomposition, so as to inhibit the thermal decomposition of PS and reduce the concentration of smoke. Therefore, the amount and rate of smoke production decreased. Therefore, the smoke production and smoke production rate are the lowest [22].

### 4.4. Corrosion Resistance and Aging Resistance of Flame Retardant PS Composite Board

Figure 6 shows the corrosion resistance and aging resistance of the flame retardant PS composite board after being immersed in 10% hydrochloric acid and 10% sodium hydroxide solution for 24 hours.

RETRACTED

It can be seen from Figure 6 that after acid-base corrosion, the performance of PS-MMH-3 has decreased to a certain extent, and the acidic environment has a great impact on the performance of PS-MMH-3. This is because some acids react with MMH, which reduces the performance of PS-MMH-3. Therefore, in the process of using materials, we need to pay attention to the acidity and alkalinity of the environment. After UV aging, the performance of PS-MMH-3 also decreased. The reason is that part of PS is aged, but the performance degradation is low due to its strong antiaging property [23, 24].

## 5. Conclusion

MMH can effectively improve the specific surface area and hydrophobicity of the material, so as to improve its dispersion in PS matrix. In PS-MMH-3, because MMH has high dispersion in PS matrix, PS-MMH-3 shows good tensile properties and elongation at break, which are 19.23 MPa and 87%, respectively.

## Figures and Tables

**Figure 1:** Setting diagram of thermal insulation wall of composite building.

**Figure 2:** Tensile strength and elongation at break of flame retardant PS composite board.

**Figure 3:** LOI values of different PS flame retardant composites.

**Figure 4:** Heat release rate of different PS flame retardant composites.

**Figure 5:** Flame retardant properties of PS composites.

**Figure 6:** Corrosion resistance and aging resistance of flame retardant PS composite board.

**Table 1:** Formula of flame retardant PS composites.

Sample	Magnesium hydroxide (MH)	Modified magnesium hydroxide (MMH)	Polystyrene (PS)
Pure PS	0	0	100
PS-MH	3	0	99
PS-MMH-1	0	1	98
PS-MMH-2	0	2	99
PS-MMH-3	0	3	97
PS-MMH-4	0	4	96

**Table 2:** Specific surface area and contact angle of MH before and after modification.

Sample	Specific surface area/(m^2^. g^−1^)	Contact angle/(°)
MH	42.671 ± 0.312	0
MMH	52.134 ± 0.124	22.6

## Data Availability

The data used to support the findings of this study are available from the corresponding author upon request.
